The article "A Rare Presentation of a Solitary Melanoma Bone Metastasis" was published in 2022. Journal: Cureus.

# A Rare Presentation of a Solitary Melanoma Bone Metastasis

**DOI:** 10.7759/cureus.21479

**Published:** 2022-01-21

**Authors:** Lucy Reipond, David Ford, Paul Cool

**Affiliations:** 1 Orthopaedic Oncology, The Robert Jones and Agnes Hunt Orthopaedic Hospital NHS Foundation Trust, Oswestry, GBR; 2 Medical Sciences, Keele University, Keele, GBR; 3 Trauma and Upper Limb, The Robert Jones and Agnes Hunt Orthopaedic Hospital NHS Foundation Trust, Oswestry, GBR

**Keywords:** palliative management, nuclear bone scan, mri- magnetic resonance imaging, computed tomography (ct ), solitary metastasis, metastasis, melanoma

## Abstract

A 74-year-old woman presented with sudden onset pain and swelling in her right wrist. Plain radiographs showed a pathological fracture through a lytic lesion. The patient had a past medical history of melanoma on her right thigh, which had been excised two years previously. She was referred to the bone cancer unit to undergo a series of investigations that included a magnetic resonance imaging scan, bone scintigraphy and a computed tomography-guided biopsy. Collectively, all investigations revealed a solitary bone metastasis from her previous melanoma in the right distal radius. The patient was treated symptomatically and underwent internal fixation with cement augmentation for symptom control. With the incidence of melanoma increasing, this case demonstrates the importance of being vigilant of unusual presentations.

## Introduction

Melanoma skin cancer is very common within the United Kingdom, with the incidence of cases increasing by 38% over the last decade [1]. Common metastatic sites of melanoma include liver, brain, intestine and bone. Bone metastases are usually found at later stages of the disease [2,3]. A solitary bone metastasis of melanoma is rare. However, with the number of cases of melanoma in the United Kingdom increasing, further research into the management of all possible presentations of the disease is needed [2]. 

## Case presentation

A 74-year-old lady presented with sudden onset severe pain and swelling in her right wrist. Two years previously she had a melanoma on her right thigh excised. Since then, she had made a full recovery and had been very well in herself. She did not have any routine surveillance appointments since, as excision of the melanoma was thought to be curative. Due to the on-going pain and swelling in her wrist, she presented to the emergency department. She was initially treated for suspected cellulitis and discharged with a course of antibiotics. However, after three weeks of continuous pain and swelling of her right wrist, she re-attended emergency department, where plain radiographs were taken.

Radiographs showed a pathological fracture through a lytic lesion within the right distal radius (Figure 1). The patient was treated with a plaster cast, analgesia and was referred to the bone cancer unit for further investigations. Investigations included a nuclear bone scan, magnetic resonance imaging (MRI) and computed tomography (CT)-guided biopsy to investigate if the lesion was primary or secondary (Figures 2, 3). Biopsy confirmed the tumour to be a metastasis from her previous melanoma (Figure 4). Complete staging was then undertaken, which included a CT scan of the chest, abdomen and pelvis. Although the bone scan indicated other areas of increased activity, they were felt to be arthritic in origin. This was also confirmed with radiographs. A CT head scan was not performed in this patient, as she did not have any symptoms or display any signs of focal neurological deficit, suggestive of brain metastases. However, there is a low threshold to undertake a CT head scan if the patient develops symptoms or signs of brain metastases. Collectively, the scans showed no further lesions, including within the viscera, confirming a solitary bone metastasis from the previous melanoma.

**Figure 1:** Plain radiographs of right arm Radiographs show a pathological fracture of the distal radius secondary to metastatic melanoma. R: right.

**Figure 2:** Nuclear bone scan The bone scintigraphy shows other areas of increased activity within the skeleton, most likely caused by arthritis as uptake is symmetrical. Unfortunately, the wrists are incompletely imaged. There is also increased uptake in the opposite left distal radius. However, radiographs of the left distal radius showed arthritic change only. L: left, R: right.

**Figure 3:** MRI of right arm MRI scan of the right distal radius, showing the metastatic lesion causing bone destruction.

**Figure 4:** Bone biopsy The biopsy of the distal radius confirmed metastatic melanoma.

Following discussion at a multi-disciplinary team (MDT) meeting, it was felt that treatment was most likely supportive rather than curative. There was a pathological fracture with significant local contamination of tumour cells, making wide local excision and reconstruction not feasible. It seemed unlikely that cure could be obtained by ablative surgery. This was discussed with the patient, and she agreed to supportive surgical treatment to improve her symptoms. The surgical aim was to reduce pain and improve function.

At surgery, the radius was approached via an anterior Henry’s approach, utilising the internervous plane between the radial and median nerves. The bone was exposed, and an intralesional curettage was performed. Subsequently, a long surgical locking plate was applied under image intensification control (Figure 5). The defect was filled and fixation augmented with Palacos® (Heraeus Medical, Newbury, United Kingdom) polymethylmethacrylate bone cement. Although the radial bone had shortened slightly, a lengthening procedure with associated risks was felt not to be appropriate, as the treatment was palliative. Further tissue was taken and submitted for histopathological review. This confirmed the pre-operative diagnosis of metastatic malignant melanoma.

**Figure 5:** Intraoperative images Intraoperative images of internal fixation of the right distal radius.

Two weeks following surgery, the patient was pain free and had an almost full range of motion in her wrist. On examination, there was no evidence of ulnar nerve impingement, and pronation and supination were full, but flexion and extension were slightly restricted to 90%. The patient was referred to clinical oncology for consideration of adjuvant radiotherapy and additional oncological treatments.

## Discussion

Management of metastatic bone tumours remains challenging. Symptomatic bone lesions require further investigation with MRI and CT scans as appropriate. An MRI allows further details of the surrounding soft tissue to be viewed, and a CT scan evaluates the bone structure better [3,4]. Even with a history of previous cancer, a solitary bone lesion should be biopsied to exclude alternative diagnoses, such as a primary bone tumour (sarcoma) and metastasis from a previously undiagnosed (other) cancer [5]. Biopsy is usually done best under image guidance, fluoroscopy or CT. Once a diagnosis of malignancy is made, complete staging should be undertaken that includes CT scan of the chest, abdomen and pelvis as well as a nuclear bone scan [3,5].

Treatment of metastatic bone disease is usually palliative. However, following further developments in oncological treatments, survival rates have improved. Particularly in solitary breast and renal metastasis, consideration should be given to complete wide excision and reconstruction, as treatment could be curative or increase the disease-free interval [5]. Unfortunately, in the majority of cases, metastatic bone disease remains incurable.

The decision regarding the correct orthopaedic treatment of metastatic bone disease can be very challenging. In the case presented, consideration was given for ablative treatment as this would be the only chance of cure. However, this was felt to be unlikely given her diagnosis and relatively short disease-free interval between diagnosis of primary and secondary tumour. Although no other metastases were identified in the investigations, further micrometastatic spread was felt to be likely.

Dormancy of melanomas has been documented in multiple studies. With some types of melanoma, tumour cells lie dormant for up to 20 years after the primary occurrence [2]. However, this is very uncommon when bone metastases have occurred. An arm amputation would give a considerable functional loss, and, on balance, it was felt that palliative surgical treatment would be the best treatment option for this patient. The treatment options were openly discussed with the patient, and she agreed to supportive treatment to control her symptoms whilst improving function.

It is also important to note that despite a palliative prognosis, it does not mean that interventions cannot be undertaken to improve quality of life. It is well known that surgical intervention of bone metastases is excellent at improving pain and restoring function [3-6]. Hence, surgery was undertaken in this case in order to try and ensure this.

The patient’s prognosis is difficult to predict. There have been many studies which analyse the mean survival period of patients with widespread metastasis, but fewer studies regarding solitary bone metastasis due to their rarer presentation. The studies that have investigated this determined that life expectancy for patients with solitary lesions compared to patients with widespread lesions is longer [3,6]. In this case, before the pathological fracture occurred, the patient was fit and well. Therefore, the status of the patient’s health, combined with the unknown prognosis, emphasised the need for surgical intervention to improve her quality of life. The aim of surgical intervention was to ensure that the patient was able to function as normal as possible, for as long as possible [3-8].

There have already been many advancements in treatments for metastatic melanomas, such as using immunotherapy targeted treatments, alongside surgical resection, chemotherapy and radiotherapy [4]. However, with the incidence of melanoma skin cancer increasing every year, continued research for different and more specific treatments to combat the disease is essential. Moreover, educating the public regarding signs of a developing melanoma and risk factors, such as increased sun exposure, remains an extremely important aspect of fighting the disease. As the earlier the disease can be caught and treated, the better the prognosis [9].

## Conclusions

In conclusion, the treatment for metastatic bone cancer remains a challenging and multifactorial branch of medicine. A series of investigations are required to confirm the bone lesion and determine its extent. Consideration should be given whether the bone lesion is a primary bone sarcoma, metastasis from a known cancer or metastasis from a new, previously undiagnosed, cancer. Solitary bone lesions usually require an image-guided biopsy for confirmation. Moreover, it is important that each individual case is discussed at an MDT meeting, ensuring that the most appropriate management is chosen for each patient. Other crucial learning points from this case include to always consider the possibility of a pathological fracture in patient with a history of sudden onset pain in their limb, without any history of trauma, especially in patients with a history of a previous cancer. Lastly, surgical intervention should still be considered and carefully planned in patients with a palliative prognosis, with the aim to improve pain and function.

A solitary bone lesion within the distal radius, secondary to a melanoma, is very rare. However, due to the increasing incidence of melanoma around the world, it raises the question if we will see more unusual presentations like this in the future.
